The article "Isolation, expression, and in silico profiling of a thermostable xylanase from Geobacillus stearothermophilus strain NASA267: insights into structural features and agro-waste valorization" was retracted in 2025. Reasons: duplicated images; overlap with earlier publications; unreliable results or conclusions; concerns about the data.

# Isolation, expression, and in silico profiling of a thermostable xylanase from *Geobacillus stearothermophilus* strain NASA267: insights into structural features and agro-waste valorization

**DOI:** 10.1186/s12934-025-02672-6

**Published:** 2025-03-21

**Authors:** Safaa M. Ali, Nehad Noby, Nadia A. Soliman, Sanaa H. Omar

**Affiliations:** 1 Nucleic Acid Research Department, GEBRI, City of Scientific Research and Technological Applications, Alexandria, Egypt; 2 Department of Biotechnology, Institute of Graduate Studies and Research, Alexandria University, Alexandria, 21526 Egypt; 3 Bioprocess Development Department, GEBRI, City of Scientific Research and Technological Applications, Alexandria, Egypt; 4 Botany and Microbiology Department, Faculty of Science, Alexandria University, Alexandria, Egypt

**Keywords:** Xylanase, Cloning, Thermal stability, TIM barrel fold, Homology model, GH10 xylanase family

## Abstract

**Background:**

Xylanase is an industrial enzyme with diverse applications, including nutritional supplements, agro-waste valorization, and paper pulp bleaching. This study aims to investigate the production of recombinant thermostable xylanase for converting plant biomass into fermentable sugars, a key step in various industrial processes.

**Results:**

*Geobacillus stearothermophilus* strain NASA267, a Gram-positive, thermophilic bacterium, was identified as the top xylanase producer from samples collected in Egypt and Saudi Arabia. The xylanase gene *xyl267* was successfully cloned from the NASA267 strain and heterologously expressed in *E. coli* under the control of a *Lambda* promoter. Optimal expression conditions were determined, with the highest enzyme activity (40 U/ml) achieved after 4 h of induction at 42 ℃. SDS-PAGE analysis revealed that the molecular weight of the recombinant xylanase was approximately 40 kDa, consistent with the calculated molecular weight (38.6 kDa) based on its amino acid sequence (331 aa). Enzyme sequence and structural analysis revealed that xyl267 shows typical TIM barrel fold where Glu134 and Glu241 constitute the enzyme active site. The xyl267 demonstrated optimal activity at 65 ℃ and maintained full stability up to 60 ℃, while it displayed a half-life of 8 min at 80 ℃. It remained stable at − 20 ℃ for up to 50 days and was most active at pH 8. Although the enzyme was active in presence of various salts, solvents, and cations, the exposure to Cu^2^⁺, Zn^2^⁺, Mn^2^⁺, and methanol reduced the enzyme activity by 47%, 37%, 31%, and 8%, respectively. The enzyme was effective in saccharifying agro-waste, particularly pretreated banana peel, which produced the highest sugar content. These findings highlight xyl267s potential for biomass conversion and industrial applications in high-temperature and alkaline environment.

**Conclusion:**

The *xyl267* from a NASA strain was cloned and successfully overexpressed in *E. coli*, producing a ~ 40 kDa recombinant enzyme. It showed optimal activity at 65 ℃, and was most active at pH 8. While it retained activity in various salts and solvents, it was inhibited by some heavy metals. Xyl267 effectively released fermentable sugars from pretreated banana peel, making it a promising candidate for industrial applications in high-temperature, alkaline environments and agro-waste saccharification.

**Supplementary Information:**

The online version contains supplementary material available at 10.1186/s12934-025-02672-6.

## Introduction

Xylan is the most abundant polysaccharide of plant hemicelluloses and the second most prevalent natural polymer after cellulose [1]. It’s a complex heterogenous polymer, consisting of different polysaccharide, including, d-galactose, l-arabinose, d-mannoses [2].

Xylanases are a group of hydrolases, capable of hydrolysing Xylan polymer into simple sugars. They belong precisely to glucoside hydrolases and can be further categorized into endo-1,4-β-xylanases, exo-1,4-β-xylanases, and α-l-arabinofuranosidases [1, 3]. Xylanases are widely applied in several industrial and biotechnological applications for example, in degrading lignocellulosic biomass, a process important in biofuel production, animal feed, paper processing [4, 5], and agricultural waste treatment. [6, 7]. In animal nutrition, xylanase-based saccharification improved broiler performance by 4–6% in feed conversion ratio and increased wheat AME (Apparent Metabolizable Energy) content by up to 6% [8, 9].

Microbial xylanases have gained wide interest in recent time. The extreme habitats of microorganism constitute a valuable source for isolating microbial enzymes of different physicochemical properties suitable for several processing conditions [10]. Thermophilic xylanases, produced by heat-tolerant organisms like *Geobacillus* [10, 11], *Thermotoga* [12], and *Bacillus* [13], are of industrial interest due to their thermostability, remaining active at high temperatures. These enzymes are suited for high-temperature industrial processes where mesophilic enzymes would lose activity [14]. Thermophilic xylanases are also resistant to thermal denaturation and maintain higher activity in harsh chemical conditions, making them versatile for industrial applications [15, 16].

Cloning and expression of xylanase genes from thermophilic bacteria have enabled the production of recombinant enzymes with enhanced properties suitable for industrial applications. Notably, the expression of thermostable xylanases in heterologous systems, such as *Escherichia coli*, has made it possible to scale up production while maintaining the enzyme’s high activity and stability [17, 18]. Advances in genetic engineering have facilitated the identification, cloning, and expression of xylanase genes from various thermophilic bacteria, such as *Geobacillus stearothermophilus* [19, 20], *Thermomyces lanuginosus* [21], and *Bacillus subtilis* [13, 22]. These species are known for their ability to produce enzymes that remain active at elevated temperatures, making them ideal candidates for industrial use.

Moreover, thermophilic bacteria possess inherent resistance to other environmental stressors,,sucj as high salinity, and extreme pH variations, which further enhances the practical utility of the xylanases they produce. By optimizing gene expression systems, such as using lambda promoters in *E. coli* or other expression vectors, researchers have successfully overexpressed thermostable xylanases at high yields, significantly improving enzyme activity and stability under various industrial conditions [23]. The successful cloning of xylanase genes has not only enhanced our understanding of their biochemical properties but also opened avenues for engineering enzymes with desired traits, such as improved thermal stability, substrate specificity, and resistance to denaturation in the presence of inhibitors or solvents [4].

This study focuses on the cloning, over-expression, and characterization of xylanase from thermophilic bacteria, exploring its potential application in agro-waste saccharification processes that require high-temperature conditions. Additionally, we perform in silico analysis of its protein structure and determine the predicted physicochemical properties of the expressed enzyme. By examining factors such as optimal induction conditions, enzyme stability, and activity under various conditions, we aim to contribute to the development of more efficient and sustainable biocatalysts for industrial applications.

## Materials and methods

### Isolation and screening of xylanase-producing thermophilic bacteria

Thermophilic and thermotolerant bacteria were isolated by incubating soil samples in LB broth at temperatures ranging from 50–70 ℃ followed by shaking at 200 rpm for 24 h. The samples were then spread on LB agar plates for single colony isolation. Pure isolates were screened for xylanase production by plating on NA agar supplemented with 0.2% (w/v) xylan. The xylan was solubilized, and 20 g/L agar was added, autoclaved, and poured into Petri dishes, which were then inoculated with the bacterial isolates. Xylanase production was qualitatively assessed by the appearance of a clear halo around colonies after staining with 0.2% (w/v) Congo red and washing with 1 M sodium chloride [24].

### Quantitative estimation of xylanase activity

Inoculations were performed by adding 1 mL of suspension from freshly prepared bacterial cultures (18 h old) into 50 mL of production medium (NA with 0.2% xylan) in 250 mL Erlenmeyer flasks. The flasks were incubated at 50 ± 2 °C for 48 h with shaking at 200 rpm. After incubation, cells were removed by centrifugation at 5000 rpm for 15 min, and the supernatant was used for enzyme activity analysis. Xylanase activity was measured by determining the amount of reducing sugars released as xylose using the dinitrosalicylic acid (DNS) method. Briefly, 0.5 mL of culture supernatant was mixed with 0.5 mL of 0.5% (w/v) birch wood xylan in 50 mM Tris–HCl buffer (pH 7.5) and incubated at 50 ℃ for 15 min. A standard curve with xylose concentrations ranging from 10–100 µg/mL was prepared, and enzyme activity was calculated. One unit of enzyme activity was defined as the amount of enzyme releasing 1 µg of xylose [25].

### Microscopic examination and molecular identification of the selected isolate

The isolate labeled NASA267, which exhibited high xylanase production, was subjected to microscopic examination using optical microscopy and scanning electron microscopy (SEM) for morphological characterization. Gram staining was performed to determine the bacterial type. Genotypic characterization was carried out by sequencing the partial *16S rRNA* gene, amplified from genomic DNA using standard PCR method. The obtained sequence was compared with database entries using BLASTn for species identification [26].

### Competent cell preparation and transformation

*E. coli* DH5α cells were used to prepare competent cells. DNA (ligation mixture) was added to the competent cells, and the mixture was incubated on ice for 20 min. Transformation was achieved by heat shock, followed by recovery in LB medium [27].

### PCR cloning of xylanase gene from *Geobacillus stearothermophilus* NASA267

The xylanase gene was amplified from the genomic DNA of *Geobacillus stearothermophilus* NASA267 using the primers F _Xyl_ 5´ATGAACAGCTCCCTCCCCT 3´ and R _Xyl_ 5´ TCAGACACTCACTGCCCTC 3´, which were designed based on conserved sequences from other thermophilic *Geobacillus* xylanase genes in NCBI GenBank (www.ncbi.nih.gov)..The software primers3 (http://bioinformatic.weizmann.acil/egibin/primer/primer3.egi) was used for primer design. The amplified PCR fragment was run on a 1% agarose gel, purified using the QIAquick Gel Extraction Kit, and cloned into the PTZ57R/T vector using the TA-cloning strategy. The ligated plasmid was transformed into *E. coli* DH5α, and colonies were screened for the presence of the insert using ampicillin -containing agar plates supplemented with IPTG (0.1 mM) and X-Gal (40 µg/ml) [28]. Positive colonies were propagated in LB medium with ampicillin (100 µg/mL), and plasmids were extracted and purified using the GeneJET Plasmid Miniprep Kit (Fermentas). The insert's size was verified by PCR using universal primers (M13F- 5´AGGCCCTGCACCTGAAG 3´& M13R- 5´TCAGCGCCTGGTACC 3´), and sequencing was performed to confirm the identity of the cloned gene.

### Sequence identity and phylogenetic analysis of xyl267

The sequence identity of the xyl267 nucleotide sequence was determined using BLASTn, and a phylogenetic analysis was conducted by aligning it with closely related sequences using ClustalW (Version 1.83). Phylogenetic analysis trees were constructed using the maximum-likelihood method in TreePuzzle (Version 5.2). The final tree was visualized using TreeView through BioEdit software (Version 6.0). Additionally, protein sequences of xylanases were retrieved from the protein database via a BLAST search using the xyl267 amino acid sequence. Multiple sequence alignments were performed, and the results were displayed in a graphical format using BioEdit software (Version 6.0).

### DNA manipulations

Chromosomal DNA, plasmid DNA, or PCR fragments were digested in a 20 μL reaction volume with 2 μL of enzyme buffer and 1–2 units of restriction enzyme (Fermentas). Ligation was carried out using T4 DNA ligase, and PCR fragments were inserted into vectors at a molar ratio of 4:1 [29].

### Construction of an active expression plasmid carrying the *xyl267 g*ene

A plasmid carrying the xylanase gene (xyl267) was constructed by PCR amplification using primers (F_Xyl_ & R_Xyl_) that included the restriction sites *Xho*I and *Sal*I, respectively. Both the expression vector (pCYTEX-P1) and the PCR product were digested with *Xho*I and *Sal*I. The resulting fragments were ligated and transformed into *E. coli* DH5α. The transformed colonies were screened for xylanase activity on LB/xylan agar plates, detected using the Congo red chromogenic agent. The constructed plasmids were sequenced using universal primers (SDM1F: 5' CCAACACTACTACGTTTTAACTGAAACAAACTGG 3' and SDM3R: 5' GCGAACGCCAGCAAGACGTAGCCCAGC 3') to confirm the cloning process.

### Heterologous overexpression of xylanase (xyl267) under the control of the Lambda promoter

To express xylanase (xyl267) in *E. coli*, 50 mL of LB ampicillin medium in 250 mL Erlenmeyer flasks was inoculated with 500 μL of overnight culture of *E. coli* DH5α carrying the pCYTEX-xyl plasmid. The culture was incubated at 37 °C with shaking at 200 rpm until the optical density (OD_600_) reached 0.7–1.0. Protein expression was induced by shifting the temperature to 42 ℃, and samples were collected at regular intervals for protein analysis and activity assays [30].

### SDS-PAGE, and zymography for xyl 267 activity detection

Protein samples (10–20 μg) were mixed with SDS-loading buffer and denatured at 95 ℃ for 5 min. The samples were then cooled on ice and loaded onto an SDS-PAGE gel. The gel was run in electrophoresis buffer for 15 min at 20 mV, followed by 3 h at 60 mV. After electrophoresis, the gel was stained and destained according to the Laemmli method [31]. To detect the active xylanase band, a zymography assay was conducted. The SDS-PAGE gel was prepared using 100 μg of protein, incubated for 1 h in a renaturation solution containing 0.5 × Triton X-100 in 50 mM phosphate buffer (pH 7.5). The renatured gel was then incubated overnight at 50 ℃ in 0.5% xylan in Tris–HCl buffer (pH 7.5, 50 mM). After incubation, the gel was transferred to a plate containing Congo red (0.005%) for 10 min and washed with 1 M sodium chloride. The appearance of a clear halo around the protein band indicated xylanase activity [32].

### Evaluation of lysis methods and lysate storage conditions

Several methods were employed to lyse *E. coli* cells expressing recombinant xylanase (xyl267). After gene induction, the cells were harvested, washed, and resuspended in 50 mM Tris buffer (pH 7.5). Lysis was achieved using three methods: chemical (1% SDS), physical (1X 1 min), and mechanical (glass beads, 0.25–0.50 mm). Enzyme activity in the cell lysate was measured every minute during the 4-min treatment using the DNS method. The most effective lysis method, based on enzyme activity, was selected for use in subsequent experiments. Additionally, the residual activity of the treated samples stored at – 20 ℃ was monitored at various time points up to 72 h.

### Optimization of induction time for xylanase (xyl267) overexpression

To optimize the induction time for xylanase (xyl267), a 50 mL culture of LB ampicillin medium was inoculated with 500 μL of overnight culture of *E. coli* DH5α carrying the pCYTEX-xyl plasmid. The culture was incubated at 37 ℃ with shaking until the OD600 reached 0.7–1.0. Protein expression was induced by shifting the temperature to 42 ℃, and samples were collected every hour for up to 30 h. The cell lysates were analyzed for enzyme activity by the DNS method.

### Enzyme homology model and structural elucidation

The homology model of xyl267 was built based on *G. stearothermophilus* 1XT6 xylanase (PDB:1N82) as a template using I-TASSER server. A multiple threading approach (LOMETS) provided by I-TASSER selects best templates based on their highest Z score. The created structural model figures were visualized using PyMOL (http:// www.pymol.org). Enzyme secondary structure analysis and active site annotation was carried out using SAS tool (https://www.ebi.ac.uk/thornton-srv/databases/sas/). Sequence variability between xyl267 and 1XT6 was carried out using Jalview 2.11.4.1 tool.

### Estimation of xyl267 physicochemical properties using *in-silico* analysis

The online server ProtParam (ExPASY) (https://www.expasy.org/resources/protparam) was used for amino acid sequence composition. Some physicochemical properties including molecular weight, pI, extinction coefficient, GRAVY (grand average of hydrophobicity), aliphatic index and instability index, in addition to statistics about protein amino acid ratios were estimated.

## Characterization of the crude recombinant xyl267

### Determination of optimal temperature

The optimal temperature for xylanase (xyl267) activity was determined over a range of 35–80 ℃ in 50 mM Tris–HCl buffer (pH 7.5).

### Determination of optimal pH

The optimal pH for xylanase activity was assessed over a pH range of 3–10 using citrate, phosphate, Tris base, and borate buffers (50 mM).

### Temperature stability

Thermal stability was evaluated by incubating the enzyme at 40–55 ℃ for up to 5 h. Additionally, stability was tested at 60 ℃, 65 ℃, 70 ℃, 75 ℃, and 80 ℃ for 10 min each with 1 min interval. Long-term stability was assessed by storing enzyme aliquots at − 20 ℃ for up to 50 days without thawing and evaluating activity after gradual thawing the stored samples.

### pH stability

The pH stability of xylanase was tested at pH 7, 7.5, 8, and 8.5 for up to 10 weeks, with the enzyme stored at − 20 ℃ throughout the experiments. Furthermore, the stability was examined at pH 8 and 8.5 at room temperature for 5 h.

### Effect of different compounds on enzyme activity

The effect of various compounds on xylanase activity was assessed by incubating the enzyme with 1 mM of chelating agents (EDTA), cations (CaCl_2_, ZnCl_2_, MgCl_2_, NaCl, MgSO_4_, MnSO_4_, FeSO_4_, CuSO_4_), and solvents (ethanol, DMSO, isopropanol, methanol, glycerol) or 0.01% SDS. After 15 min of incubation, residual enzyme activity was measured and compared to untreated controls to determine the effect of each compound on enzyme activation or inhibition.

### Agro-waste saccharification using recombinant xyl267

This experiment utilized various types of agro-waste materials, including rice straw, banana peel, sawdust, newsprint, filter paper, and dried plant residues. The samples were first dried overnight at 60 ℃ in an oven, then ground into a powdered form. A 1% sample of each material was tested individually. The testing process began by mixing the waste materials with 1 ml of 1% NaOH solution and incubating the mixture at room temperature for 4 h, afterward, the samples were autoclaved for 20 min. The pretreated materials were then neutralized by adding HCl to counteract the alkali, and they were subsequently used as substrates for enzyme saccharification. For the saccharification process, 200 U of recombinant xyl267 enzyme dissolved in Tris–HCl buffer (pH 8.0) was added to the pretreated materials. The enzyme solution was filtered through a bacterial filter (0.2 µm) before being added to the substrate mixture. The mixture was incubated with mild shaking at 50 ℃, and the production of reducing sugars was measured daily using the DNS method, with glucose as the standard [30]. The total reducing sugar production from both pretreated and untreated waste materials was monitored over a two-week period and compared.

### Statistical analysis

The data were plotted using Excel software version 4 and presented as the mean ± standard error from three replicate samples for each test.

## Results

### Screening and identification of thermostable xylanase-producing bacteria

A screening program was conducted to isolate thermostable xylanase-producing bacteria from Egypt and Saudi Arabia. Among the selected strains in total 226, NASA267 showed the highest xylanase production and was identified as *Geobacillus stearothermophilus* through *16S rRNA* sequencing (Accession No. KC788496.1), where it showed 99.86% identity to *Geobacillus stearothermophilus* strain mt-10 (Accession No. EU652081.1). Microscopic examination confirmed that NASA267 is a Gram-positive bacterium with a short rod shape (Fig. 1). This strain was chosen for further experimentation due to its promising enzyme production and thermophilic nature.

**Fig. 1:** Microscopic examination of strain NASA267: Ligt microscope image (left), Scanning electron microscope image (right)

### Cloning of the xylanase gene (xyl267)

The xylanase gene (*xyl267*) from *Geobacillus stearothermophilus* NASA267 was cloned using PCR with the F_xyl_ and R_xyl_ primers, which amplified a ~ 1000 bp fragment. The PCR product was purified, inserted into the PTZ57R/T vector via TA-cloning, and transformed into *E. coli* DH5α. The TA-cloning strategy and clone verification are shown in Fig. 2. Successful clones were identified by the white colony color, and plasmids were extracted from these positive colonies. The presence and size of the insert were confirmed by PCR and sequencing. BLASTn analysis revealed that the insert shared 97.41% identity with the *Geobacillus* sp. Y412MC52 complete genome (Accession No. CP002442.1) (Table 1S), specifically the coding sequence for *Endo-1,4-beta-xylanase*. A phylogenetic tree was constructed based on the translated amino acid sequence of xyl267, incorporating the closest related sequences, as shown in Fig. 3. The analysis clearly indicates that xyl267 clusters with endo-1,4-beta-xylanases from *Geobacillus thermopakistaniensis, Geobacillus* and *Geobacillus stearothermophilus* (Accession No. ESU73079.1, WP_013523887.1 & AAZ74783.1), respectively.

**Fig. 2:** Schematic diagram illustrating the TA-cloning strategy used for the PCR product obtained with primers (xyl_F_ and xyl_R_) to amplify the xylanase gene

**Fig. 3:** Phylogenetic analysis of the *xyl267* gene from the bacterial *Geobacillus stearothermophilus* strain NASA267, compared to other bacterial xylanases available in the GenBank database. The dendrogram was generated using the neighbor-joining method in BioEdit software. The following abbreviations were used: *G. thermopak* (*Geobacillus thermopakistaniensis*), *G. stearother* (*Geobacillus stearothermophilus*), *G. thermodeni* (*Geobacillus thermodenitrificans*), *Parabeobac* (*Parabeobacillus*), *Baci* (*Bacillus*), *uncul* (uncultured), *Evan cellu* (*Evansella cellulosilytica*), *Caldicellu saccha* (*Caldicellulosiruptor saccharolyticus*), *Caldicellu kran* (*Caldicellulosiruptor kronotskyensis*), and *Segni roi* (*Segniliparus rotundus*)

### Phylogenetic analysis of the cloned xyl267

A consensus coding sequence of the *xyl267* gene (996 bp) was obtained, and its amino acid sequence (331 aa) (Fig. 1S) was compared to NCBI GenBank data using BLAST. It showed 92.79% identity to the *endo-1,4-beta-xylanase* gene of *Geobacillus* sp*.* (Accession No. ESU73079.1 & WP_013523887.1) (Table 2S). For phylogenetic analysis, multiple sequence alignments were performed using ClustalW. A graphical view of the aligned sequences revealed the presence of two conserved Glu residues in the enzyme active site across the aligned sequences, as shown in the supplementary figure (Fig. 2S).

### Heterologous expression of *xyl267* gene in *E. coli*

The xylanase gene (xyl267) from *Geobacillus stearothermophilus* NASA267 was successfully expressed using the pCYTEX-P1 expression vector. Primers with *Xho*I/*Sal*I restriction sites were designed to clone the gene under the lambda promoter. The full subcloning procedure is summarized in the supplementary diagram (Fig. 3S). After subcloning the target gene, transformants were screened for xylanase activity on LB ampicillin and xylan agar plates using Congo red. Active clones, identified by the appearance of a halo zone after induction at 42 ℃, were selected, and plasmids were extracted. PCR and restriction digestion confirmed the presence of the target gene in the plasmids, as shown in Fig. 4. The intracellular activity of recombinant proteins from clones 1, 2, and 3 was tested after sonication using the DNS method and plate assay (Fig. 5). Clone number 3 demonstrated the highest activity and was selected for further experimentation.

**Fig. 4:** Stepwise selection for the best recombinant clone carrying the *xyl267* xylanase gene from *Geobacillus stearothermophilus* strain NASA267

**Fig. 5:** Activity verification of recombinant *xyl267* clones (1, 2, & 3) using the qualitative plate assay method (**A**) and the quantitative DNS method (**B**) to assess enzyme activity

### Optimization of cell lysis method for recombinant xyl267 expression

Recombinant xyl267 was overexpressed in *E. coli* DH5α under the lambda promoter by shifting the temperature to 42 ℃. The cells were cultured in LB-ampicillin medium at 37 ℃ with shaking at 200 rpm. After 6 h of induction (OD_600_ ~ 1.0), cell pellet was collected and subjected to lysis using three different methods: SDS treatment, sonication, and glass bead disruption. Intracellular enzyme activity was monitored every minute during the lysis process (Tables 3S). The results indicated that sonication for 1 min yielded the highest enzyme activity (36 U/ml), followed by SDS treatment for 3 min and glass bead disruption for 4 min, which both resulted in 29 U/ml activity. When the lysates were stored at − 20 ℃, sonication preserved stable or nearly complete enzyme activity for up to 72 h, outperforming the other methods (Table 4S). Based on these results, sonication was chosen as the method for use in subsequent experiments.

### Expression analysis of recombinant *xyl267* under *Lambda* promoter

Xyl267 expression was monitored at various induction times (0–4 h) using a temperature shift from 37 to 42 °C. Protein samples from these time points were quickly analyzed via SDS-PAGE and in situ activity staining. The activity stain revealed a prominent band around 40 kD (Fig. 6). Further expression analysis, focusing on activity, was conducted on samples collected over a 30-h induction period and is shown in Fig. 7. The highest activity (40 U/ml) was observed after 4 h of induction, which was determined to be the optimal time.

**Fig. 6:** SDS-PAGE and zymogram analysis of recombinant xyl267 enzyme production upon induction. The induced active xyl267 enzyme band (~ 40 kDa) is clearly visible, indicated by the arrow. M: protein marker (left side, stained with Coomassie Brilliant Blue stain); zymogram (right side). Lane 0: pre-induction (zero time); Lanes 1–4: samples taken after 1, 2, 3 & 4 h after induction, respectively

**Fig. 7:** Optimal induction time for recombinant xyl267 enzyme production

### Sequence analysis and structural elucidation of xyl267 enzyme

The homology model of xyl267 xylanase was built based on the 3D structure of IXT6 xylanase from *G. stearothermophilus* (PDB 1N82), with an identity 92% and Z score 5.

Sequence analysis of xyl267 in comparison to other homologs shows a two conserved Glu residues (Glu 134, Glu 241) found opposite to each other on loop 3 and β sheet 7, respectively, constituting the enzyme active site (Figs. 8, 9A). The structural analysis of xyl267 shows a TIM-barrel fold (α/β)_8_ with a salad bowel form, representative to GH10 enzymes (Fig. 9B). The surface topology shows a deep cleft at the centre of the structure, for accommodating large polymer (Fig. 9C). Sequence alignment between xyl267 and 1XT6 template showed sequence difference at the C terminal region (Fig. 10A). The 3D Structural alignment between xyl267 xylanase and IXT6 displayed a root mean square deviation (RMSD) with 0.243 (Fig. 10 B).

**Fig. 8:** Sequence annotation of xyl267 illustrating its secondary structure elements using SAS software from Expasy

**Fig. 9:** Overall structure and active site representation of *xyl267.* The typical (β/α)₈ barrel fold is shown, with α-helices in cyan and β-strands in magenta. The catalytic triad residues, Glu134 and Glu241, are highlighted in green (**A**). A side view of the ribbon diagram illustrating the “salad-bowl” shape, a characteristic feature of GH10 family members (**B**). The surface topology of the enzyme, revealing an extended groove suitable for accommodating polymeric substrates, consistent with its endo-mode of action (**C**)

**Fig. 10:** Sequence variability between *xyl267* and IXT6 in the C-terminal region (Helix 8 and Loop 8) illustrated with Jalview software (**A**). 3D structural alignment of *xyl267* (yellow) and IXT6 (cyan), with an RMSD of 0.243 (**B**)

### Estimation of the physicochemical properties of xyl267 using in silico analysis

The predicted molecular weight of xyl267 xylanase is 38.65 kDa, and its theoretical isoelectric point (pI) is 5.76, indicating an acidic nature for the enzyme. Theoretically, a pI value below 7 further confirms the acidic character of the protein. The enzyme exhibits a high aliphatic index of 81.9 and a negative GRAVY value, suggesting favorable hydrophilic properties. The instability index indicates that the protein has low stability. Leucine, glutamine, and aspartate are the predominant amino acids in the xyl267 sequence. Table 1 summarizes the predicted physicochemical parameters of xyl267.

**Table 1:** The predicted physicochemical parameters of xyl267 enzyme

Parameters	Xyl267
Molecular Weight (Da)	38,651.10
Theoretical pI	5.76
Extinction coefficient (M^–1^ cm^–1^)	57,410
Instability index	42.58
Aliphatic index	81.9
Grand average of hydrophobicity (GRAVY)	-0.389
Number of negatively charged amino acids (Asp + Glu)	50
Number of positively charged amino acids (Arg + Lys)	39
Predominant amino acids	
Leucine	8%
Aspartate	7.6%
Glutamine	7.6%

## Characterization of the crude recombinant xyl267 enzyme

### Effect of temperature

As described in materials and methods different temperatures (35–85 ℃) were tested to determine the optimal value. The data plotted and shown in Fig. 11A, where it was noticed that, concerning xyl267 the optimal value appeared at 65 ºC.

**Fig. 11:** Optimum temperature of the recombinant xyl267 enzyme activity (**A**) and thermostability of recombinant xyl267 enzyme at temperatures ranging from 60 to 80 ℃ (**B**)

To determine the thermal stability of the tested enzyme, the residual activities of the xyl267 enzyme were recorded against time exposure for each temperature 35, 40, 45, 50, 55, 60, 65, 70, and 75 ℃. The xyl267 enzyme showed total stability at 35 and 40 ℃ for 4 h, at 45 and 50 ℃ stable for 2.5 h, at 55 and 60 ℃ stable for 90 min. A noticeable drop in thermal stability for the *xyl267* enzyme was recognized by raising the temperature to 65, 70, 75, and 80 ℃, where the xylanase enzyme lost 26, 40, 48, and 54% after 10 min exposure, respectively as shown in Fig. 11B. The enzyme’s half-life was approximately 8 min at 80 ℃.

### Effect of freezing at − 20 ℃

The stability of the recombinant xyl267 enzyme was tested at − 20 ℃ for up to 50 days, with and without thawing. Under conditions of no thawing, the enzyme remained completely stable throughout the 50-day period. However, when subjected to gradual thawing, the enzyme retained stability for approximately 30 days, losing about 35% of its activity after 50 days, as shown in Fig. 12.

**Fig. 12:** Effect of freezing at − 20 ℃ with grudal thawing on recombinant xyl267 enzyme activity

### Effect of pH

The crude recombinant xyl267 enzyme activity rate was studied as a function of pH ranging from 5 to 10. Figure 13A, demonstrated that, xyl267 has a great preference for working in an alkaline condition where the optimum was recorded at pH 8.

**Fig. 13:** Optimum pH for recombinant xyl267 enzyme activity (**A**) and monitoring the pH stability of recombinant *xyl267* enzyme activity during long-term preservation at − 20 ℃, without thawing (**B**)

The stability of the recombinant xyl267 enzyme was tested after preservation at different pH levels (7, 7.5, 8, and 8.5) under cooling conditions (− 20 ℃) for 10 weeks, as illustrated in Fig. 13B. The enzyme remained stable, with only a slight loss (12%) in activity at pH 8.5. Further, the stability was tested at pH 8 and 8.5 at room temperature for 5 h, during which the enzyme exhibited full stability throughout the duration (data not shown).

### Effect of different compounds

The effect of various cations, solvents, SDS, and glycerol on the activity of the crude xyl267 enzyme was investigated. The results demonstrated that the presence of MgCl_2_, MgSO_4_, CaCl_2_, NaCl, FeSO_4_, EDTA, DMSO, ethanol, isopropanol, glycerol, and SDS did not reduce enzyme activity. In contrast, exposure to CuSO_4_, ZnCl_2_, MnSO_4_, and methanol led to a decrease in enzyme activity by 47%, 37%, 31%, and 8%, respectively (Fig. 14).

**Fig. 14:** Effect of different substances on recombinant *xyl267* enzyme activity [3]

### Saccharification of agro-waste materials using recombinant xyl267 enzyme

As shown in Table 5S, the highest total reducing sugars (approximately 176 mg/L) were produced from pretreated banana peel after 7 days of treatment with crude recombinant (*xyl267)* xylanse enzyme. Overall, the pretreatment of agro-waste materials enhanced the catalytic action of the *xyl267* enzyme, resulting in increased sugar release from all tested materials. The lowest amount of reducing sugars (58 mg/L) was obtained from rice straw, which contains recalcitrant compounds, particularly lignin, that are difficult to degrade. In contrast, more predictable sugar yields were observed from other materials: sawdust (100 mg/L), filter paper (79 mg/L), plant residues (64 mg/L), and newspapers (60 mg/L).

## Discussion

In this study, a systematic approach was employed to isolate and identify thermostable xylanase-producing bacteria from Egypt and Saudi Arabia. Among the strains isolated, NASA267, identified as *Geobacillus stearothermophilus*, exhibited the highest xylanase production and was selected for further characterization and experimentation. The successful isolation of this strain underscores the potential of thermophilic bacteria from diverse geographical regions for industrial enzyme production, particularly xylanases that are crucial for applications in biofuel production, food processing, and paper industries due to their ability to degrade hemicellulose [4]. The use of *16S rRNA* sequencing has become a powerful tool for establishing phylogenetic and evolutionary relationships among organisms [33]. Phylogenetic analysis, supported by sequence comparisons, facilitates the classification and grouping of genera and species, providing insights into their interrelatedness according to conventional taxonomic methods [34]. In the case of NASA267, the *16S rRNA* sequence analysis revealed that the isolate is closely related to *Geobacillus stearothermophilus*, with a 99.86% identity, confirming its affiliation with this species.

The cloning of the *xyl267* gene from *Geobacillus stearothermophilus* NASA267 involved the use of PCR amplification, TA-cloning, and transformation into *E. coli* DH5α, resulting in successful recombinant clones. The cloned gene showed a high degree of similarity (92.79%) to the *Endo-1,4-beta-xylanase* gene from *Geobacillus* species, supporting the accuracy of the gene identification and the evolutionary proximity of these strains [35].

Heterologous expression of the *xyl267* gene in *E. coli* DH5α successfully demonstrated enzyme production under the lambda promoter system. Induction of the recombinant protein was achieved by shifting the temperature to 42 °C, which is consistent with previous studies on the overexpression of thermophilic lipase in *E. coli* DH5α under the lambda promoter [36], as well as thermophilic α-amylase in the pET-SUM system using *E. coli* BL21 (DE3) host cells [37]. Additionally, the pCYTEXP1 expression vector, which utilizes the λ promoter, has been effectively employed for overexpressing thermophilic carboxyl esterase, resulting in higher yields of active enzyme [38]. Esterases from *B. subtilis* and *B. stearothermophilus* were also cloned and expressed in *E. coli* using an L-rhamnose expression system, yielding greater quantities of active enzyme compared to expression in *B. brevis* [39]. Screening for xyl267 activity on xylan agar plates identified clone number 3 as having the highest enzyme activity, which was confirmed by quantitative enzyme assay. These findings suggest that this recombinant *E. coli* clone is capable of producing significant levels of active xylanase, which is a crucial step for scaling up enzyme production for industrial applications.

Optimization of the cell lysis method revealed sonication as the most effective approach for releasing recombinant xylanase, yielding the highest enzyme activity. This method not only ensured high protein yield but also preserved enzyme activity over time, making it a reliable technique for enzyme extraction. This is consistent with other studies that report sonication as an efficient means for cell disruption in recombinant protein production, particularly for membrane-bound or intracellular enzymes [20, 40].

The expression of recombinant xyl267 under the control of the lambda promoter was successfully monitored through SDS-PAGE and in situ activity staining, allowing for the tracking of both protein production and enzymatic activity. The prominent induced band observed at approximately 40 kDa corresponds to the expected molecular weight of the xylanase enzyme, confirming the successful expression of the xyl267 recombinant protein. The molecular weight of the enzyme (xyl267) is consistent with other xylanases reported in the literature. For instance, *Bacillus* sp. strain NG-27 [10], *Geobacillus* sp. strain DUSELR13 [41], and *Caldicoprobacter algeriensis* [42] produce xylanase enzymes with molecular weights of 42 kDa, ~ 45 kDa, and 52 kDa, respectively. In addition, studies on the genetic manipulation of xylanase-producing microorganisms have revealed that *Bacillus tequilensis* BT21, isolated from marine sediments, produces an extracellular xylanase. The *xynBT21* gene encoding the enzyme was successfully cloned and expressed in *E. coli*, resulting in a protein of 213 amino acids and a calculated molecular mass of 23.3 kDa [43].

The expression investigation of xyl267 over a 30-h induction period revealed that the highest enzymatic activity (40 U/ml) was achieved after 4 h of induction at 42 °C. This information is essential for scaling up enzyme production in future applications, where maximizing both yield and activity is essential. Also, this result suggests that the *Lambda* promoter in *E. coli* is highly effective in driving xyl267 expression at the chosen temperature. The observed peak in activity at 4 h likely corresponds to the maximal synthesis of the xylanase enzyme and accumulation of active enzyme in the cells. The noticed decline in activity after 4 h of induction could be attributed to the saturation of the expression system or the instability of the enzyme at higher expression levels, which may lead to protein degradation or misfolding. This is consistent with findings in other studies where optimal enzyme activity is observed within a narrow induction window, and overexpression beyond this period can result in decreased yields of functional enzyme [44–46].

Sequence analysis and 3D structural modeling revealed that xyl267 belongs to the family 10 xylanases, similar to the structural template 1XT6 xylanase, which was used to build the enzyme's homology model. Despite high sequence similarity (92%), the sequence alignment between xyl267 and 1XT6 showed variations in the C-terminal region, specifically at loop 8 and helix 8. The N- and C-terminal regions are known to influence protein folding and enzyme stability. Many studies have demonstrated that mutations in these regions can enhance enzyme thermal stability [47]. This suggests that exploring the physicochemical properties of both enzymes based on C-terminal variability could lead to further improvements in enzyme stability.

Thermostable xylanases offer significant advantages in lignocellulosic conversion. Conducting reactions at high temperatures accelerates the hydrolysis process by enhancing the solubility of both reactants and products. Additionally, high temperatures disrupt the biomass cell wall structure, which improves enzyme accessibility and overall efficiency of the conversion process [48, 49].

The enzyme’s activity (xyl267) was stable under a range of temperatures, with optimal activity at 65 ℃, making it a promising candidate for industrial applications that require thermostable enzymes [50]. This result aligns with xylanases from thermophilic organisms, which typically show optimal activity at higher temperatures. For example, the optimum temperatures for xylanases from *Geobacillus* sp. strain DUSELR13, *Trichoderma harzianum* strain, the recombinant thermostable endo-xylanase from alkalophilic, mesophilic *Bacillus* sp*.* strain NG-27, recombinant xylanases from *Bacillus sonorensis* T6, recombinant xylanase from alkaliphilic thermophilic *Bacillus* sp*.* NCIM59, and GH10 xylanase from *Caldicellulosiruptor bescii* are 75 ℃, 65 ℃, 70 ℃, (47–55 ℃), 60 ℃, and 70 ℃ [10, 13, 22, 42, 51, 52], respectively. In contrast, xylanases from mesophilic organisms such as *Bacillus subtilis* VSDB5 and *Bacillus licheniformis* KBFB4 exhibit optimal activity at lower temperatures, typically around 50 ℃ [53].

The thermal stability of the enzyme (xyl267) was evaluated across a range of temperatures, revealing exceptional stability between 35 and 50 ℃, where it maintained significant activity over prolonged periods. This suggests its potential effectiveness in industrial applications requiring moderate thermal conditions. At 55 and 60 ℃, the enzyme remained stable for 1.5 h before activity declined significantly. At temperatures between 65 and 80 ℃, activity decreased by 26%, 40%, 48%, and 54%, respectively, after 10 min of exposure, with a half-life of 8 min at 80 °C, highlighting the typical instability of proteins at extreme thermal conditions. Notably, the enzyme’s ability to retain activity at temperatures up to 60 ℃ for extended periods further underscores its potential for industrial applications, especially in high-temperature environments. So, the xyl267 enzyme exhibits moderate thermostability, with an instability index of 42.58 predicted by in silico analysis using the Portparam server, which aligns with experimental results indicating low protein stability for values above 40. For comparison the xylanase from *Geobacillus* sp*.* strain DUSELR13 exhibits exceptional thermostability, with half-lives of 48, 38, and 13 days at 50, 60, and 70 ℃, respectively [10]. The xylanase from *Trichoderma harzianum* remains stable at 65 ℃ for 4 h [51]. The xylanase from *Thermomyces lanuginosus* VAPS24 maintains stability at 80 ℃ for 60 min [54], while the recombinant xylanase from *Bacillus* sp. NCIM59 retains 100% activity at 50 ℃ for 24 h and has a half-life of 2 h at 60 ℃ [13]. The xylanase from *Caldicellulosiruptor bescii* (GH10) shows a half-life of approximately 7.7 h at 60 ℃ [52]. The enzyme from the thermophilic fungus *Myceliophthora heterothallica* retains over 50% activity after 1 h at 65 ℃ and about 30% activity after 1 h at 70 ℃ [55]. Additionally, recombinant xylanases from *Caldicoprobacter algeriensis* and *Bacillus* sp. strain NG-27 exhibit half-lives of 20 min at 80 ℃ and 30 min at 70 ℃, respectively [41, 42]. The xylanases from *Bacillus subtilis* VSDB5 and *Bacillus licheniformis* KBFB4 retain 40% of their activity after 30 min at 60 ℃ [53].

Thus, although the xyl267 enzyme exhibits moderate thermostability, it compares favourably with other xylanases, especially in terms of its stable activity at moderate temperatures, which is beneficial for various industrial applications. The observed reduction in activity at higher temperatures is typical for enzymes, as structural denaturation commonly leads to diminished functionality [56].

Enzyme hydrophobicity plays a crucial role in enzyme thermal stability, as hydrophobic interactions help maintain a more compact structure, thereby enhancing stability at elevated temperatures. It has been reported that 80.2% of the analyzed thermophilic proteins exhibit a higher degree of hydrophobicity compared to mesophilic proteins [57]. The GRAVY (Grand Average of Hydrophobicity) value indicates the relative hydrophobicity or hydrophilicity of a protein’s amino acid sequence. For example, the negative GRAVY value of xyl267 suggests that the protein is non-polar [58]. Further insight into the enzyme’s hydrophobic nature can be gained by examining the predominant amino acids in its sequence. In the case of xyl267, hydrophobic residues such as Leu, Ile, and Val are the most abundant.

The aliphatic index is another parameter that helps explain enzyme thermal stability. It reflects the volume occupied by the aliphatic side chains of Ala, Val, Ile, and Leu. This index is considered a positive factor contributing to the increased thermostability of proteins [59]. The aliphatic index of xyl267 is 81.65, compared to 56.29 for two thermostable xylanases, VSDB5 and KBFB4 from *Bacillus subtilis* VSDB5 and *Bacillus licheniformis* KBFB4 [53]. This difference in aliphatic index can help explain the higher thermal stability of xyl267.

The enzyme’s stability at − 20 ℃ was tested over a 50-day period, with xyl267 maintaining stability for up to 30 days. After 50 days, approximately 35% of its activity was lost. This suggests that the enzyme retains a reasonable degree of stability during long-term storage, making it suitable for freezing conditions. This stability is comparable to that of proteins from thermophilic bacteria, which generally exhibit good stability in freezing conditions. However, some loss of activity over extended periods is inevitable due to the rigidity effects caused by ice disrupting the enzyme’s native conformation [60].

Further investigation into the pH stability of the recombinant xyl267 enzyme revealed optimal activity at pH 8, which aligns with its preference for alkaline conditions. This characteristic is particularly advantageous for industrial applications such as paper and biofuel production, where alkaline environments are commonly encountered [61]. The enzyme also demonstrated good stability across a range of alkaline pH values, further enhancing its industrial potential. Many xylanases from thermophilic organisms exhibit optimal activity at higher pH levels, reflecting the conditions in which these organisms thrive. For instances, the endo-xylanase from Alkalophilic *Bacillus* sp. strain NG-27 is active at pH 8.4 [42]. The enzyme's sustained stability at room temperature across pH 8 and 8.5 further underscores its suitability for practical applications. It has been reported that an enzyme's optimal activity and stability at high pH can be attributed to the ratio of charged residues, with enzymes that have a higher ratio of negatively charged amino acids functioning well under alkaline conditions. Xyl267 has a negative-to-positive charged amino acid ratio of 1.28, which is higher than that of 1B30 (0.96) from *Penicillium simplicissimum*, which displays optimal activity at pH 5.6 [62]. In contrast, the 2UWF xylanase from *Bacillus halodurans* S7 has an even higher ratio of 1.67, with an optimal pH of 9–9.5 [63].

Regarding compatibility with various compounds, the enzyme xyl267 maintained robust activity in the presence of several salts: MgCl_2_, MgSO_4_, CaCl_2_, NaCl, FeSO_4_, solvents: ethanol, isopropanol, SDS, EDTA and glycerol, which is advantageous for use in diverse processing environments. However, exposure to heavy metals such as Cu^2^⁺, Zn^2^⁺, and Mn^2^⁺ resulted in a reduction in enzyme activity by 47%, 37%, and 31%, respectively, indicating potential inhibitory effects. The sensitivity of xyl267 to these metal ions may be due to their binding to the enzyme, which interferes with its activity. The presence of methanol also led to a minor decrease in enzyme activity (8%), suggesting that xyl267 could be used in environments where these compounds are present at low concentrations. These findings underscore the importance of optimizing reaction conditions and identifying suitable co-factors to enhance enzyme stability and activity in industrial processes [64]. In comparison to other xylanases, the xylanase from *Geobacillus* sp. strain DUSELR13 exhibited increased activity with the addition of Cu^2^⁺, Zn^2^⁺, K⁺, and Fe^2^⁺ at 1 mM concentration, and Ca^2^⁺, Zn^2^⁺, Mg^2^⁺, and Na⁺ at 10 mM concentration [10]. Similarly, the xylanase from *Trichoderma harzianum* showed enhanced activity with Fe^2^⁺, Mg^2^⁺, and Zn^2^⁺. However, metal ions such as Hg^2^⁺, Fe^2^⁺, Cu^2^⁺, and reagents like PEG-2000 and EDTA were inhibitory [51], while Zn^2^⁺, Na⁺, K⁺, and β-mercaptoethanol acted as activators for xylanase activity in *T. lanuginosus* VAPS24 [54]. The GH10 xylanase from *Caldicellulosiruptor bescii* was stable in the presence of some detergents and organic solvents, while *Cohnella* sp*.* A01 xylanase remained stable in the presence of various detergents and organic solvents as well [52, 65], respectively.

Highlighting the effectiveness of the recombinant xyl267 enzyme in saccharifying various pretreated agro-waste materials, it was found that pretreated banana peel produced the highest amount of reducing sugars (176 mg/L), suggesting that it is an efficient substrate for xylanase-mediated hydrolysis.. This is in line with previous studies showing that alkaline pretreatment, such as NaOH, enhances the accessibility of cellulose and hemicellulose by breaking down lignin [66]. Rice straw, however, yielded the lowest amount of reducing sugars (58 mg/L), likely due to its high lignin content, which makes it more resistant to enzymatic degradation [67]. This confirms the challenge of hydrolyzing lignin-rich materials, as lignin’s protective effect on cellulose and hemicellulose limits enzyme action [68]. Other materials, such as sawdust, filter paper, plant residues, and newspapers, produced intermediate sugar yields, indicating that *Xyl267* can effectively hydrolyze hemicellulose from these substrates. The variability in sugar yields emphasizes the importance of material selection and pretreatment optimization for efficient saccharification. The use of the DNS method to measure reducing sugars provided a reliable approach to monitor saccharification progress [30]. These results highlight the potential of recombinant *xyl267* for biomass conversion, though further optimization may be necessary for more recalcitrant materials like rice straw.

## Conclusion

In conclusion, this study demonstrates the successful isolation, characterization, and expression of a thermostable xylanase (xyl267) from *Geobacillus stearothermophilus* NASA267, highlighting its potential for various industrial applications. The recombinant xylanase exhibited optimal activity at 65 °C and maintained substantial stability at moderate temperatures, making it an attractive candidate for industries requiring high-temperature processing. Despite some reduction in activity at higher temperatures, the enzyme's performance under conditions ranging from pH 8 to 8.5 further supports its industrial viability, particularly in biofuel, paper, and food processing applications. Additionally, the enzyme’s robustness in the presence of salts, solvents, and certain metals suggests its adaptability to diverse processing environments. The successful enzyme production and efficient saccharification of agro-waste materials such as banana peel underscore its potential in biomass conversion, though further optimization of substrate pretreatment and reaction conditions is needed to enhance its performance with more recalcitrant materials. These findings provide valuable insights into the application of recombinant xylanases for industrial biotechnology and set the stage for future studies to refine enzyme performance and maximize yields for large-scale processes.

## Supplementary Information

Additional file 1.

## Data Availability

All data generated or analysed during this study are included in this article. No datasets were generated or analysed during the current study.
